# Exosomal TAR DNA binding protein 43 profile in canine model of amyotrophic lateral sclerosis: a preliminary study in developing blood-based biomarker for neurodegenerative diseases

**DOI:** 10.1080/07853890.2022.2153162

**Published:** 2022-12-10

**Authors:** Penelope Pfeiffer, Joan R. Coates, Yajaira M. Esqueda, Andrew Kennedy, Kyleigh Getchell, Myra McLenon, Edina Kosa, Abdulbaki Agbas

**Affiliations:** a Kansas City University, Kansas City, MO, USA; b University of Missouri-Columbia, Columbia, MO, USA; c Heartland Center for Mitochondrial Medicine, Kansas City, KS, USA

**Keywords:** TDP-43, amyotrophic lateral sclerosis, degenerative myelopathy, exosome, biomarker

## Abstract

**Objective:**

Blood-based biomarkers provide a crucial information in the progress of neurodegenerative diseases with a minimally invasive sampling method. Validated blood-based biomarker application in people with amyotrophic lateral sclerosis would derive numerous benefits. Canine degenerative myelopathy is a naturally occurring animal disease model to study the biology of human amyotrophic lateral sclerosis. Serum derived exosomes are potential carriers for cell-specific cargoes making them ideal venue to study biomarkers for a variety of diseases and biological processes. This study assessed the exosomal proteins that may be assigned as surrogate biomarker that may reflect biochemical changes in the central nervous system.

**Methods:**

Exosomes were isolated from canine serum using commercial exosome isolation reagents. Exosomes target proteins contents were analyzed by the Western blotting method.

**Results:**

The profiles of potential biomarker candidates in spinal cord homogenate and that of serum-derived exosomes were found elevated in dogs with degenerative myelopathy as compared to control subjects.

**Conclusions:**

Serum-derived exosomal biomolecules can serve as surrogate biomarkers in neurodegenerative diseases.

**KEY MESSAGES**
- A canine with degenerative myelopathy can serve as a model animal to study human amyotrophic lateral sclerosis.
- Serum-derived exosomes contain Transactive Response DNA Binding Protein 43 (TDP-43), a potential biomarker candidate.
- The levels of spinal cord TDP-43 proteins and that of serum-derived exosomes exhibited similar profiling. Therefore, serum derived exosomes may be used as a venue for establishing blood-based biomarkers for neurodegenerative diseases.

## 1. Introduction

The aberrant protein aggregation in motor neurons is the hallmark of amyotrophic lateral sclerosis (ALS). ALS is a progressive disease that directly affects motor neurons, leading to loss of muscle function. About 5–10% of the inherited forms of ALS are linked to a mutation in the SOD1 gene (*SOD1*). The misfolded mutant [Cu/Zn] superoxide dismutase (SOD1) protein is believed to contribute to the development of ALS, yet the role of misfolded non-mutant SOD1 in the disease progress is unclear. Recently, chemically modified aberrant Transactive Response DNA Binding Protein 43 (TDP-43) species were found to represent a major accumulating protein in neuronal cytoplasmic inclusions [1,2] and in exosomes [3,4] in Frontotemporal Lobar Degeneration (FTLD), and in ALS patients [5]. Exosomes are nano-size membranous vesicles that contain several macromolecules including aberrant pathological proteins [6]. The size and membranous structure of exosomes allow them to pass through the blood–brain barrier [7–9]. These features make exosomes a potential platform in which targeted biomolecules can be analyzed.

The biomolecular link and clinical similarities between human ALS and canine degenerative myelopathy (DM) suggested that human ALS hallmark signature proteins (i.e. SOD1 and TDP-43) have the same or similar profile in canine DM. These similarities may be employed to further biomarker validity studies such as reproducibility, specificity, sensitivity, and robustness. As a naturally occurring disease in the pet population, canine DM has many similarities to human ALS and is thought to be a result, in part, of mutated SOD1 protein in dogs. Thus, dogs affected with DM can serve as an animal disease model for ALS based on CNS size and complexity, and disease characteristics.

ALS is an incurable and fatal disease with a patient survival rate of 3–5 years once diagnosed [10]. In most patients, the symptoms begin in the lower limbs [11,12]. Patients often complain of tripping, stumbling, foot drop, or a ‘slapping’ gait. Upper limb involvement includes decreased dexterity in the fingers, cramping, stiffness, weakness, and wrist drop [13]. Early diagnosis of ALS is very difficult, which can delay the time to treatment [14]. Establishing a blood-based biomarker(s) will help clinicians with early diagnosis and initiating timely treatment. The pharmaceutical intervention with well-timing may improve the quality of life and lifespan for ALS patients.

ALS researchers have used rodents as an animal model with mutated SOD1 to study the pathology of the disease [15]. The rodent model is of limited use as disease progression is very short (3–6 months) and is based on overexpression of the human gene for mutant SOD1. In addition, peripheral biomarker studies are difficult to perform in a longitudinal course due to limited access to serial samples of serum/exosomes in mice due to the small volume of blood. Canine DM is a late adult neurodegenerative disease accompanied by (*SOD1*) mutations (*SOD1:c.118A, SOD1:c52T*), and protein aggregation [16,17]. Early clinical signs include general proprioceptive ataxia and spastic upper motor neuron paresis in the pelvic limbs with progression to flaccid tetraplegia and dysphagia [18–20]. DM and ALS are characterized by progressive multisystem neurodegeneration involving upper and lower motor neurons. Canine DM phenotypically resembles upper motor onset ALS in reference to clinical and histopathologic features. The distribution of lesions and clinical disease progression in DM are similar to that reported for the UMN-onset ALS [21] with UMN signs in DM-affected dogs progressing later to LMN signs [16,20].

An abnormal accumulation of TDP-43 has been demonstrated in the cytoplasm and platelets of ALS patients [22]. The post-translationally modified derivatives of TDP-43 (i.e. hyper-phosphorylation and ubiquitination) have been studied in ALS [23,24]. Prior research has established that the accumulation of TDP-43 in the cytosol was causal in the loss of function in affected neurons [25,26]. However, the percent of TDP-43 in peripheral blood, which represents the central nervous system (CNS) origin of TDP-43, is unknown. Therefore, assessment of the confined TDP-43 in exosomes may reflect the changes in TDP-43 protein better than that of the large volume of serum or plasma where the target proteins are diluted. This study explored the feasibility of using exosomes to assess potential biomarkers for DM such as TDP-43, pTDP-43, and SOD1.

## 2. Materials and methods

### 2.1. Animals

Previously −80 °C frozen spinal cord tissues from the thoracic region and serum samples were obtained from Dr. Joan R. Coates at the College of Veterinary Medicine, University of Missouri-Columbia under the approval of the institutional animal care and use committee (IACUC# 10077). Pet owners signed an informed consent for samples being used for research purposes.

Whole blood was collected from the jugular or cephalic veins. Blood was centrifuged and serum was placed in 500 μL aliquot tubes. Aliquots were stored at −80 °C. The dog was necropsied for CNS tissue collections. The muscle was removed from the dorsal column of the spine. The dorsal lamina just medial to the articular processes was removed to expose the spinal cord. Specifically, the thoracic spinal cord was removed and sectioned accordingly. The tissues were immediately frozen on dry ice and stored at −80 °C.

Tissues were harvested from various breeds with diagnosed DM and age-matched dogs not affected with DM (Table 1 in Supplemental Data). All DM affected dogs were homozygous for the SOD1 E40K mutation [20].

### 2.2. Isolation of exosomes from canine serum

The isolation of exosomes from the serum of DM and control dogs was performed using a commercially available particle precipitation method following the manufacturer’s protocol (miRCURY Exosome Serum/Plasma Kit, Qiagen #76603). The exosome isolation procedure was based on the capture of water molecules, which otherwise would form the hydrate envelope of particles in suspension. Mixing the starting sample with a proprietary precipitation buffer diminished the hydration of the subcellular particles and allowed the precipitation of even particles smaller than 100 nm with a low-speed centrifugation step [27]. Before proceeding to the isolation of exosomes, the serum samples were first pelleted by centrifugation, and the supernatant was filtered through 0.20-μm filtration disk to remove residual cells, debris, platelets, large micro vesicles, etc. The samples were incubated with a proprietary precipitation buffer for 1 h at 4 °C. After a 30-min low speed centrifugation at 500 × *g*, the exosomes pellets were re-suspended for further analysis of their content. The isolated exosomes were verified by immunoprobing assay using an antibody that recognized exosome surface protein, tumor susceptibility 101 protein (TSG101) (Supplemental Figure 3). Exosome suspension was aliquoted and kept in −20 °C until use.

### 2.3. Spinal cord homogenate preparation

Fifty to 60 mg thoracic spinal cord tissue (T3 section) was homogenized in an ice-cold buffer (0.32 M sucrose, 0.5 mM MgSO_4_, 10 mM ε-amino-n-caproic acid, protease inhibitor cocktail (0.05% v/v) (Calbiochem #539134), phosphatase inhibitor cocktails set II (0.1% v/v) (Calbiochem # 524625), 10 mM HEPES, pH 7.4) in a glass pestle-glass homogenizer (8–10 strokes). The tissue/homogenization buffer ratio was one (mg tissue)/15 (µL buffer). The homogenate was resuspended 8–10 times using a 1 mL syringe with a 26-gauge needle to shear DNA and liberate nuclear proteins. The homogenate was incubated on ice for 20 min and subjected to centrifugation at 16,000 × *g* for 20 min at 4 °C. The supernatant containing all soluble proteins, including nuclear proteins was collected into a clean tube. For purpose of the protein assay, 5–10 µL aliquot was saved. Total protein estimation was analyzed by BCA assay (ThermoFisher Scientific #23225). The sample was aliquoted into 100 µL volumes into microfuge tubes and stored at −80 °C until use.

### 2.4. Immunoblotting analysis

Ten micrograms of exosomal proteins were loaded onto a commercial 4–20% SDS/PAG gradient gel. The electrophoresis was run at 100 V for 75–80 min until the dye-front migrated to 0.5 cm from the bottom of the gel. Resolved proteins on the gel were transferred onto a PVDF membrane by electro transfer unit at 60 V for 90 min. The membrane was stained/destained for total protein staining according to the manufacturer’s protocol (REVERT Total Protein Stain kit, LI-COR; Cat# 926-11016). The membrane was blocked with a blocking agent (SEA BLOCK Blocking, Thermo Scientific, Cat # UH2788881) for 1 h at room temperature, followed by overnight incubation with anti- TDP-43 Ab (1:1000 dilution; Proteintech Cat# 10782-2-AP), anti-P(S409/410) TDP-43 Ab (1:1000 dilution; Proteintech Cat# 66318-1-Ig), and anti-SOD1 Ab (1:750 dilution; Proteintech Cat#10269-1-AP) on an orbital shaker at 4 °C. The next day the membrane was incubated with Infrared (IR)-tagged antibody (1:10,000 dilution; LI-COR Cat# 926-3211, 926-68071, 926-32210, 926-68070) for 1–2 h at room temperature. The protein bands were visualized in an image analyzer (LI-COR Odyssey Infrared Imager (Model No. 9120). The band intensity was normalized based on total protein staining signals, and analyzed by Image Studio image analyzing program (V.3.1, Li-COR Biosciences).

## 3. Results

### 3.1. Dogs with DM spinal cord homogenate show elevated TDP-43 and SOD1 in the thoracic region of the spinal cord

The thoracic region of the spinal cord from companion dogs with DM (*n* = 4) and from age matched non-DM affected control dogs (*n* = 4) were obtained from a tissue archive at the University of Missouri College of Veterinary Medicine. The signalment of dogs used in this study listed in Table 1 in Supplemental Data. Figure 1 shows that TDP-43 protein levels are elevated in the DM spinal cord region as compared to that of the control dogs. A *t*-test analysis indicated that differences between the two groups were significant (*p* < 0.01). This observation agrees with other published data that TDP-43 accumulation has been observed in the human spinal cord [23,28]. SOD1-immunoreactive aggregates were observed in ventral horn motor neurons [29]. This study confirmed that the spinal cord SOD1 aggregation profile occurred in dogs with DM (Figure 2). In this study, the SOD1 aggregation profile was considered as positive control.

**Figure 1.** Total TDP-43 levels of thoracic region of spinal cord homogenate. TDP-43 levels were elevated in the spinal cord homogenate from DM affected dogs (*n* = 4, Supplemental Data/Table 1: dog # 1,2,3,4) as compared to that of the control dogs (*n* = 4, Supplemental Data/Table 1: dog # 5,6,7,8) [One-sample *t*-test (**p < 0.01)]. The protein band intensity were normalized to total protein staining.

**Figure 2.** SOD1 levels of thoracic region of spinal cord homogenate. SOD1 levels were elevated in the spinal cord homogenate from DM affected dogs (*n* = 4, Supplemental Data/Table 1: dog # 1,2,3,4) as compared to that of the control dogs (*n* = 4, Supplemental Data/Table 1: dog # 5,6,7,8) [One-sample *t*-test (**p < 0.01)]. The protein band intensities were normalized to total protein staining.

### 3.2. Exosomal TDP-43, phosphorylated TDP-43, and SOD1 are elevated in canine with DM

Frozen serum samples from dogs were obtained from a tissue archive at the University Of Missouri College Of Veterinary Medicine. The signalments of dogs used in this study were listed in Tables 2 and 3 in Supplemental Data. Figures 3(A,B) showed that both total TDP-43 and its phosphorylated derivative (pTDP-43) were elevated in exosomes of the dogs affected with DM as compared to that of the control dogs. A significant difference (*p* ≤ 0.001) was found between DM affect and control dogs. These preliminary results suggest that exosomes can be used to assess biomarker proteins such as TDP-43 and its phosphorylated derivatives.

**Figure 3.** Serum derived exosomal total TDP-43 and phosphorylated TDP-43 profile in DM affected dogs. Both total TDP-43 (A) and phosphorylated TDP-43 (pTDP-43) (B) levels were elevated in serum-derived exosomes from DM affected dogs (*n* = 12; Table 2/Supplemental Data: dog # 1,2,3,4,5,6,7,8,9,10,11,12) compared to control dogs (*n* = 10; Table 3/Supplemental Data: dog# 1,2,3,4,5,6,7,8,9,10). One-sample *t*-test analysis revealed statistical significance for total TDP-43 (****p < 0.0001) and for pTDP-43 (***p < 0.001) Original immunoblot analysis pertinent to this figure provided in Supplemental Figures 1 and 2. The protein band intensities were normalized to total protein staining.

Serum-derived exosomal SOD1 protein levels were elevated in dogs affected with DM as compared to that of control dogs. The difference between the two groups was significant based on an unpaired *t*-test analysis (*p* ≤ 0.05). We have observed that SOD1 proteins in canine serum-derived exosomes exhibited a heterogenic profile (i.e. monomer, trimer, and tetramer) (Figure 4). Soluble monomers (∼25 kDa) were considered in the data analyses and graphing.

**Figure 4.** Serum derived exosomal SOD1 profile in dogs with DM; (A) Exosomal SOD1 levels appear to be elevated in dogs with DM. The difference between control (*n* = 3, Table 3/Supplemental Data; dog #1,2,4,5) and DM (*n* = 4; Table 2/Supplemental Data: dog #1,2,3,4,6) groups did achieve statistically significance (*p < 0.05). (B) Monomer SOD1 proteins bands were analyzed and graphed. The protein band intensities were normalized to total protein staining.

## 4. Discussion

The complexity of a biosample matrix and the invasive nature of tissue sampling led investigators to develop peripheral tissue-based biomarkers for ALS. Blood-based biomarker initiatives have gained popularity due to easy access for sampling with minimal invasion (i.e. venous puncture), access to several blood cells, and subcellular structures. Once developed and validated, blood-based biomarkers will be utilized for diagnosis, monitoring the prognosis, and monitoring the treatment of ALS [30–32].

Canine degenerative myelopathy (DM) is an adult-onset, progressive neurodegenerative disease that shares important similarities to ALS including clinical presentation and progression, pathological features, and *SOD1* mutations [33]. This naturally occurring disease in the companion dog recapitulates some forms of human mutant SOD1 ALS. The E40K SOD1 mutation is widespread among companion dogs [34] and leads to SOD1 aggregate accumulations within cells, the putative mechanism of disease in DM, and in both familial and sporadic forms of human ALS [16,35–37].

In this preliminary study, we demonstrated that serum-derived exosomes may be utilized for assessing ALS hallmark proteins (i.e. TDP-43, pTDP-43, and SOD1), and compared to that of thoracic spinal cord homogenate in DM affected dogs. We chose the thoracic region because the disease pathology of canine DM is most severe in this region [33]. This region also reflects more TDP-43 accumulation relevant to pathology of ALS [38]. Serum exosomes were isolated from the dog cohort consisting of animals with DM and age-matched non-DM affected. Due to some technical obstructions and limited tissue amount, we were unable to isolate sufficient exosomes from the spinal cord tissue from this cohort. We are currently refining our techniques to increase the exosome yield.

This study demonstrated the feasibility of the followings: (i) effectively isolating exosomes from serum, (ii) analyze exosomal TDP-43 and pTDP-43 protein profiles, and (iii) comparing those profiles to spinal cord tissue (thoracic region) homogenate from the different cohort of dogs with DM as part of proof- of- concept studies. TDP-43 and SOD1 are known as the hallmark proteins for ALS [23,24,39]. This study demonstrated that total homogenates of spinal cord TDP-43 levels were elevated in dogs with DM (Figure 1). The SOD1 profile served as a positive control and established that both proteins were elevated (Figure 2). The next logical step would be to demonstrate sensitivity and specificity to establish biomarker reliability within the study limitations due to the lack of the biosample archive that did not follow the specified minimal information for studies of extracellular vesicles, MISEV2018 [40].

Exosomes are small stable single-membrane organelles that carry selected proteins, lipids, nucleic acids, and glycoconjugates [6]. Exosome biogenesis is a valuable mechanism to assess the protein quality control [6]. They are emerging as key mediators of communication and waste management among neurons, glial cells, and connective tissues during normal and diseases conditions [41]. Although exosomes are being developed as therapeutic agents in multiple disease models, they can also serve as surveillance agents by transporting aberrant proteins like hyper-phosphorylated TDP-43 or cytosolic TDP-43 that accumulates in cell plasma. Using the dog DM model may establish the link between the spinal cord and serum/plasma-derived exosomes in terms of TDP-43 biochemistry. We have observed increased TDP-43 and SOD1 levels in exosomes derived from DM affected dog. SOD1 analysis was performed to further confirm the spinal cord and serum exosome crosstalk in terms of the content TDP-43 and its derivative.

The SOD1 protein profile revealed three SOD1 species (monomer, trimer, and tetramer), although SOD1 resolved under the reducing conditions. Recent observations demonstrated that trimer-SOD1 aggressively promoted cell death [42,43]. Because of their small size, exosomes can easily pass the blood–brain barrier to serve as accessible biomarkers of neuronal dysfunction [7,9,44,45]. This pilot study provided some preliminary data to support the notion that spinal cord TDP-43 may be transported *via* exosomes, and that TDP-43 loaded exosomes appear in the blood. However, we did not perform spinal cord-derived exosomal TDP-43 and SOD1 assessments. Hence, we do not claim yet serum-derived exosomal TDP-43 and SOD1 directly reflecting that of spinal cord. Studies are undergoing to further isolate spinal cord-derived exosomes that appeared in serum and analyze their cargo content in terms of TDP-43 and SOD1.

The concept of serum-derived exosome analysis for potential biomarker candidates will eliminate very invasive tissue and cerebrospinal fluid sampling and allows investigators to obtain repeated blood samples with a minimal invasive sampling method for exosome isolation. Exosomes derived from serum represent global exosomes which include neuronal derived exosomes (NDE) [46]. A recent review has discussed on astrocyte-derived extracellular vesicles in the blood may be a useful tool for detecting astrocyte-specific biomarkers in neurological conditions [47,48]. Our current research is focusing on the development of a process, to selectively isolate the NDE population from global serum and spinal cord tissue-derived exosomes.

The availability of a disease model that more closely reflects the human condition would provide an opportunity to test if the pathologic processes shown to contribute to the motor neuron disease in rodent models are likely to contribute to ALS. Such a model could also be used in second-generation preclinical trials to shield ALS patients from participation in clinical trials with little probability of success. In addition, studies with the proposed disease model may reveal disease processes that are shared with the ALS cases but do not occur or are difficult to detect, in the rodents due to small size, short lifespan, or other issues. Ideally, the desired disease model would develop both upper and lower motor neuron signs due to a single spontaneous mutation in an orthologue of a human gene known to harbor ALS-causing mutations. This model would involve an animal species that is intermediate between rodents and humans in life expectancy and in the size and complexity of the CNS. It would be readily available on a wide variety of genetic backgrounds negating the need to maintain research colonies. It would display a disease phenotype that, similar to ALS, first manifests in mature individuals. In addition, the initial clinical signs would consistently appear at the same anatomic site and spread throughout the body in a uniform in pattern and rate. Canine DM has all these features and is therefore another disease model for understanding ALS. Companion dogs with DM represent a clinical population confounded by complexities in diagnosis, comorbidity, and environmental and genetic diversity similar to those encountered in a human clinical trial setting. Thus, the incorporation of veterinary clinical trials into the ALS treatment development paradigm will enhance translational efficiency by identifying and optimizing those therapies most likely to generate clinical benefit.

## Data Availability

The authors confirm that the data supporting the findings of this study are available within the article and its Supplementary Materials. The data are available on reasonable request from corresponding author (aagbas@kansascity.edu).

## References

[1] Beyer L, Gunther R, Koch JC, et al. TDP-43 as structure-based biomarker in amyotrophic lateral sclerosis. Ann Clin Transl Neurol. 2021;8(1):271–277.33263951 10.1002/acn3.51256PMC7818221

[2] Majumder V, Gregory JM, Barria MA, et al. TDP-43 as a potential biomarker for amyotrophic lateral sclerosis: a systematic review and meta-analysis. BMC Neurol. 2018;18(1):90.29954341 10.1186/s12883-018-1091-7PMC6027783

[3] Iguchi Y, Eid L, Parent M, et al. Exosome secretion is a key pathway for clearance of pathological TDP-43. Brain. 2016;139(Pt 12):3187–3201.27679482 10.1093/brain/aww237PMC5840881

[4] Hosaka T, Yamashita T, Tamaoka A, et al. Extracellular RNAs as biomarkers of sporadic amyotrophic lateral sclerosis and other neurodegenerative diseases. Int J Mol Sci. 2019;20(13):3148.10.3390/ijms20133148PMC665112731252669

[5] Suk TR, Rousseaux MWC. The role of TDP-43 mislocalization in amyotrophic lateral sclerosis. Mol Neurodegener. 2020;15(1):45.32799899 10.1186/s13024-020-00397-1PMC7429473

[6] Pegtel DM, Gould SJ. Exosomes. Annu Rev Biochem. 2019;88:487–514.31220978 10.1146/annurev-biochem-013118-111902

[7] Saint-Pol J, Gosselet F, Duban-Deweer S, et al. Targeting and crossing the blood–brain barrier with extracellular vesicles. Cells. 2020;9(4):851.32244730 10.3390/cells9040851PMC7226770

[8] Morad G, Carman CV, Hagedorn EJ, et al. Tumor-derived extracellular vesicles breach the intact blood–brain barrier via transcytosis. ACS Nano. 2019;13(12):13853–13865.31479239 10.1021/acsnano.9b04397PMC7169949

[9] Qu M, Lin Q, Huang L, et al. Dopamine-loaded blood exosomes targeted to brain for better treatment of Parkinson’s disease. J Control Release. 2018;287:156–166.30165139 10.1016/j.jconrel.2018.08.035

[10] What is ALS? The ALS Association; 2014 [updated 2014 Feb 16]. Available from: www.alsa.org

[11] Wijesekera LC, Leigh PN. Amyotrophic lateral sclerosis. Orphanet J Rare Dis. 2009;4:3.19192301 10.1186/1750-1172-4-3PMC2656493

[12] Turner MR, Brockington A, Scaber J, et al. Pattern of spread and prognosis in lower limb-onset ALS. Amyotroph Lateral Scler. 2010;11(4):369–373.20001488 10.3109/17482960903420140PMC3182546

[13] Masrori P, Van Damme P. Amyotrophic lateral sclerosis: a clinical review. Eur J Neurol. 2020;27(10):1918–1929.32526057 10.1111/ene.14393PMC7540334

[14] Armon C. Amyotrophic lateral sclerosis. Medscape; 2014. Available from: http://emedicine.medscape.com/article/1170097-overview

[15] Wegorzewska I, Baloh RH. TDP-43-based animal models of neurodegeneration: new insights into ALS pathology and pathophysiology. Neurodegener Dis. 2011;8(4):262–274.21124004 10.1159/000321547PMC3214943

[16] Awano T, Johnson GS, Wade CM, et al. Genome-wide association analysis reveals a SOD1 mutation in canine degenerative myelopathy that resembles amyotrophic lateral sclerosis. Proc Natl Acad Sci USA. 2009;106(8):2794–2799.19188595 10.1073/pnas.0812297106PMC2634802

[17] Holder AL, Price JA, Adams JP, et al. A retrospective study of the prevalence of the canine degenerative myelopathy associated superoxide dismutase 1 mutation (SOD1:c.118G > A) in a referral population of German Shepherd dogs from the UK. Canine Genet Epidemiol. 2014;1:10.26401327 10.1186/2052-6687-1-10PMC4579386

[18] Morgan BR, Coates JR, Johnson GC, et al. Characterization of intercostal muscle pathology in canine degenerative myelopathy: a disease model for amyotrophic lateral sclerosis. J Neurosci Res. 2013;91(12):1639–1650.24043596 10.1002/jnr.23287PMC4096151

[19] Morgan BR, Coates JR, Johnson GC, et al. Characterization of thoracic motor and sensory neurons and spinal nerve roots in canine degenerative myelopathy, a potential disease model of amyotrophic lateral sclerosis. J Neurosci Res. 2014;92(4):531–541.24375814 10.1002/jnr.23332PMC4096142

[20] Coates JR, Wininger FA. Canine degenerative myelopathy. Vet Clin North Am Small Anim Pract. 2010;40(5):929–950.20732599 10.1016/j.cvsm.2010.05.001

[21] Gordon PH, Cheng B, Katz IB, et al. Clinical features that distinguish PLS, upper motor neuron-dominant ALS, and typical ALS. Neurology. 2009;72(22):1948–1952.19487653 10.1212/WNL.0b013e3181a8269b

[22] Sage J, Hall L, McVey A, et al. Use of capillary electrophoresis immunoassay to search for potential biomarkers of amyotrophic lateral sclerosis in human platelets. J Vis Exp. 2020;156(e60638):1–9.10.3791/6063832090995

[23] Neumann M, Kwong LK, Lee EB, et al. Phosphorylation of S409/410 of TDP-43 is a consistent feature in all sporadic and familial forms of TDP-43 proteinopathies. Acta Neuropathol. 2009;117(2):137–149.19125255 10.1007/s00401-008-0477-9PMC2693625

[24] Neumann M, Sampathu DM, Kwong LK, et al. Ubiquitinated TDP-43 in frontotemporal lobar degeneration and amyotrophic lateral sclerosis. Science. 2006;314(5796):130–133.17023659 10.1126/science.1134108

[25] Baloh RH. TDP-43: the relationship between protein aggregation and neurodegeneration in amyotrophic lateral sclerosis and frontotemporal lobar degeneration. FEBS J. 2011;278(19):3539–3549.21777387 10.1111/j.1742-4658.2011.08256.xPMC3177991

[26] Jo M, Lee S, Jeon YM, et al. The role of TDP-43 propagation in neurodegenerative diseases: integrating insights from clinical and experimental studies. Exp Mol Med. 2020;52(10):1652–1662.33051572 10.1038/s12276-020-00513-7PMC8080625

[27] miRCURY Exosome kits handbook. Qiagen; 2017. p. 7–8. HB-2434-001_1107923_HB_miRCURY_Exo_Isolation_Kits_1217%20(3).pdf

[28] Feneberg E, Charles PD, Finelli MJ, et al. Detection and quantification of novel C-terminal TDP-43 fragments in ALS-TDP. Brain Pathol. 2021;(4):e12923.10.1111/bpa.12923PMC841207433300249

[29] Katz ML, Jensen CA, Student JT, et al. Cervical spinal cord and motor unit pathology in a canine model of SOD1-associated amyotrophic lateral sclerosis. J Neurol Sci. 2017;378:193–203.28566164 10.1016/j.jns.2017.05.009

[30] Sun J, Carrero JJ, Zagai U, et al. Blood biomarkers and prognosis of amyotrophic lateral sclerosis. Eur J Neurol. 2020;27(11):2125–2133.32557963 10.1111/ene.14409

[31] Aydemir D, Ulusu NN. Importance of the serum biochemical parameters as potential biomarkers for rapid diagnosis and evaluating preclinical stage of ALS. Med Hypotheses. 2020;141:109736.32315925 10.1016/j.mehy.2020.109736

[32] Brodovitch A, Boucraut J, Delmont E, et al. Combination of serum and CSF neurofilament-light and neuroinflammatory biomarkers to evaluate ALS. Sci Rep. 2021;11(1):703.33436881 10.1038/s41598-020-80370-6PMC7803734

[33] Averill DR Jr. Degenerative myelopathy in the aging German Shepherd dog: clinical and pathologic findings. J Am Vet Med Assoc. 1973;162(12):1045–1051.4196853

[34] Zeng R, Coates JR, Johnson GC, et al. Breed distribution of SOD1 alleles previously associated with canine degenerative myelopathy. J Vet Intern Med. 2014;28(2):515–521.24524809 10.1111/jvim.12317PMC4238831

[35] Rakhit R, Chakrabartty A. Structure, folding, and misfolding of Cu, Zn superoxide dismutase in amyotrophic lateral sclerosis. Biochim Biophys Acta. 2006;1762(11–12):1025–1037.16814528 10.1016/j.bbadis.2006.05.004

[36] Forsberg K, Jonsson PA, Andersen PM, et al. Novel antibodies reveal inclusions containing non-native SOD1 in sporadic ALS patients. PLOS One. 2010;5(7):e11552.20644736 10.1371/journal.pone.0011552PMC2904380

[37] Bosco DA, Morfini G, Karabacak NM, et al. Wild-type and mutant SOD1 share an aberrant conformation and a common pathogenic pathway in ALS. Nat Neurosci. 2010;13(11):1396–1403.20953194 10.1038/nn.2660PMC2967729

[38] Noto Y, Shibuya K, Sato Y, et al. Elevated CSF TDP-43 levels in amyotrophic lateral sclerosis: specificity, sensitivity, and a possible prognostic value. Amyotroph Lateral Scler. 2011;12(2):140–143.21126161 10.3109/17482968.2010.541263

[39] Neumann M, Kwong LK, Truax AC, et al. TDP-43-positive white matter pathology in frontotemporal lobar degeneration with ubiquitin-positive inclusions. J Neuropathol Exp Neurol. 2007;66(3):177–183.17356379 10.1097/01.jnen.0000248554.45456.58

[40] Thery C, Witwer KW, Aikawa E, et al. Minimal information for studies of extracellular vesicles 2018 (MISEV2018): a position statement of the International Society for Extracellular Vesicles and update of the MISEV2014 guidelines. J Extracell Vesicles. 2018;7(1):1535750.30637094 10.1080/20013078.2018.1535750PMC6322352

[41] Song Z, Xu Y, Deng W, et al. Brain derived exosomes are a double-edged sword in Alzheimer’s disease. Front Mol Neurosci. 2020;13:79.32547364 10.3389/fnmol.2020.00079PMC7274346

[42] Zhu C, Beck MV, Griffith JD, et al. Large SOD1 aggregates, unlike trimeric SOD1, do not impact cell viability in a model of amyotrophic lateral sclerosis. Proc Natl Acad Sci USA. 2018;115(18):4661–4665.29666246 10.1073/pnas.1800187115PMC5939103

[43] Proctor EA, Fee L, Tao Y, et al. Nonnative SOD1 trimer is toxic to motor neurons in a model of amyotrophic lateral sclerosis. Proc Natl Acad Sci USA. 2016;113(3):614–619.26719414 10.1073/pnas.1516725113PMC4725519

[44] Saeedi S, Israel S, Nagy C, et al. The emerging role of exosomes in mental disorders. Transl Psychiatry. 2019;9(1):122.30923321 10.1038/s41398-019-0459-9PMC6438960

[45] Banks WA, Sharma P, Bullock KM, et al. Transport of extracellular vesicles across the blood–brain barrier: brain pharmacokinetics and effects of inflammation. Int J Mol Sci. 2020;21(12):4407.10.3390/ijms21124407PMC735241532575812

[46] Malm T, Loppi S, Kanninen KM. Exosomes in Alzheimer’s disease. Neurochem Int. 2016;97:193–199.27131734 10.1016/j.neuint.2016.04.011

[47] Upadhya R, Zingg W, Shetty S, et al. Astrocyte-derived extracellular vesicles: neuroreparative properties and role in the pathogenesis of neurodegenerative disorders. J Control Release. 2020;323:225–239.32289328 10.1016/j.jconrel.2020.04.017PMC7299747

[48] Long X, Yao X, Jiang Q, et al. Astrocyte-derived exosomes enriched with miR-873a-5p inhibit neuroinflammation via microglia phenotype modulation after traumatic brain injury. J Neuroinflammation. 2020;17(1):89.32192523 10.1186/s12974-020-01761-0PMC7082961

